The article "Reinforcement of Self-Regulated Brain Activity in Schizophrenia Patients Undergoing Rehabilitation" was published in 2021. Journal: Biomed Res Int.

# Reinforcement of Self-Regulated Brain Activity in Schizophrenia Patients Undergoing Rehabilitation

**DOI:** 10.1155/2021/8030485

**Published:** 2021-03-26

**Authors:** Renata Markiewicz, Beata Dobrowolska

**Affiliations:** ^1^Psychiatric Nursing Department, Faculty of Health Sciences, Medical University of Lublin, 20-081 Lublin, Poland; ^2^Department of Management in Nursing, Faculty of Health Sciences, Medical University of Lublin, 20-081 Lublin, Poland

## Abstract

The experiment was aimed to compare the effects of different forms of rehabilitation applied in patients with schizophrenia. Verification of the obtained results was based on the analysis of the level of cognitive and social functioning of the subjects. For this purpose, the following clinical tools were used: Positive and Negative Syndrome Scale (PANSS), Beck Cognitive Insight Scale (BCIS), Color Trial Test (CTT-1, CTT-2), d2 psychological tests, Acceptance of Illness Scale (AIS), Self-efficacy Scale (GSES), Quantitative Electroencephalogram Biofeedback (QEEG-BF), auditory event-related potentials (ERPs), and serum levels of brain-derived neurotrophic factor (BDNF). The subjects were mentally stable male schizophrenia patients who had been in remission. They were divided into two groups which received different types of rehabilitation for three months. Group 1 patients followed a standard rehabilitation and Group 2 patients received GSR Biofeedback (*galvanic skin response Biofeedback, GSR-BF*) training. Pretherapy and posttherapy measurements were made for each group. Experimental rehabilitation based on GSR-BF training resulted in regulatory control of neurophysiological mechanisms, and the parameters obtained demonstrated improvement in the subjects' cognitive and social function. The following therapy outcomes were observed: (1) reduce psychopathological symptoms (2) improving cognitive (concentration, attention) and social functions (3) increase in the neurotrophic factor BDNF. GSR-BF can be used as an alternative to conventional rehabilitation in schizophrenia patients.

## 1. Introduction

Schizophrenia is a disease with a multifactorial pathogenesis and a recurrent course [1]. The long-term disease process leads to severe cognitive and executive deficits. These dysfunctions are associated with disturbances in the function of various brain regions [2], mainly the frontal and temporal regions, limbic and midline brain structures, and basal ganglia [1, 3, 4], which lead to impairments in working memory, concentration, emotions and everyday functional outcomes [1, 5–10].

Schizophrenia, as a disease with a variable course, requires multidirectional treatment that includes both pharmacotherapy and rehabilitation. There are different forms of therapy, amongst which Biofeedback (BF) is gaining in popularity. More and more studies confirm the positive effect of BF therapy in people diagnosed with anxiety disorders [11, 12], depression [13–16], bipolar disorder [17, 18], and schizophrenia [19, 20].

Depending on the type of brain–computer interface (BCI) used, various forms of BF are distinguished. In the present therapeutic experiment, we used galvanic skin response BF (GSR-BF).

GSR has two components, the general tonic-level electrodermal component (skin conductance level, SCL) and the phasic component (skin conductance responses, SCR_S_), which are indispensable diagnostic parameters in the management of mental disorders. They can be used as references in GSR-BF to modulate the patient's emotional state depending on the current needs [21]. The ability to reduce stress presumably increases the patient's sense of coherence, protects them against relapse, enhances their cognitive processes, and improves their quality of life.

Currently, there are few publications that explore this topic, but it seems worth investigating given the compensatory capacities of the nervous system, i.e., its plasticity, which occurs at many levels and is conditioned by external influences. In this light, BF training can be viewed as a form of external influence which uses specific exercises to modify the structure and function of neural networks through learning and memorizing. Regular training results in dynamic reorganization of synapses and neuronal expression of genes, including BDNF. Together with other proteins, BDNF is involved in neuronal function [22–27], growth and differentiation of stem cells, formation of synapses, regulation of neuronal circuits [27], and the formation of memory pathways [26, 28, 29]. BDNF is expressed when neurons are active, i.e., when energy processes and the associated changes in potential occur. Under the influence of these processes, neurotransmitters are produced, which enable the remodeling of the synaptic network and the formation of new connections. Synaptic reorganization occurs when changes in action potential are induced by effective stimulation [29–32], such as GSR BF training.

In order to verify the assumptions made in the study and to verify the effect of therapy based on the GSR-BF method, two groups of patients, men with a clinical diagnosis of schizophrenia, in remission, were compared in which two different forms of rehabilitation were applied: standard rehabilitation (Group 1) vs. GSR-BF training (Group 2).

## 2. Materials and Methods

The convenience sample of mentally stable male schizophrenia patients who had been in remission for the past 1.5 years and continued treatment with atypical neuroleptics. The subjects were divided into two groups. Group 1 (26 individuals) included patients who followed a conventional rehabilitation program, and Group 2 (18 individuals) was comprised of patients undergoing GSR-BF training. Both groups received rehabilitation for three months.

The following instruments were used in the study:

1. The Color Trails Test (CTT) of cerebral dysfunction: part 1 (CTT-1)—to assess visual performance and psychomotor speed, and part 2 (CTT-2)—to assess performance skills and working memory [33]
2. The d2 test of attention—to measure processing speed (amount of material processed in a specific time), quality of work (accuracy and the errors made), and persistence as an indicator of features of behaviour manifested during work (irritation, stability of work or lack of it—discouragement, fatigue) [34]
3. PANSS, a scale evaluating psychopathological symptoms of schizophrenia [35]
4. The Beck Cognitive Insight Scale (BCIS) [36]
5. The Acceptance of Illness Scale (AIS) [37]
6. The Self-efficacy Scale (GSES) [37]
7. QEEG-BF amplitudes and frequency ratios [38]

Neuropsychological assessment was performed by a psychologist, and BDNF levels were determined by a laboratory diagnostician (Serum BDNF levels were determined by the immunoenzymatic technique ELISA (Human BDNF ELISA kit, R&D Systems, Minneapolis, MN, USA).

### 2.1. Patient Inclusion Criteria and Training Procedure

The subjects were recruited from among patients of a day psychiatric ward. They were informed about the therapy and the study. The inclusion criteria for patients to take part in the study were their consent, male gender (in order to eliminate hormonal differences) [39], age within the range of 18-50 years, and clinical diagnosis of schizophrenia without active or past neurological diseases, being in remission (in a stable mental state without psychotic (productive) symptoms, for minimum 1.5 years before taking part in a study). The exclusion criteria were lack of patient's consent to take part in the study, mental disability, dementia, and alcohol addiction. Patients who gave their consent and met the inclusion criteria had been set the training schedule.

All patients took atypical neuroleptics, both before entering the study and during treatment. Any change in treatment and exacerbation of mental health problems were the reasons for excluding individuals from the study.

The GSR-BF training sessions were conducted in the CENTER (relaxation), BALANCE (concentration), and INSECTS (self-control) modules using a Digi-Track apparatus (Elmiko-Medical Company, Warsaw, Poland), whose validity and accuracy of measurements was verified by the so-called validity passport (calibration 1/year) while maintaining the same external testing conditions (climatic conditions of the room where the training took place). The detailed procedure of training was described in a study already published, showing results obtained in a Group 2 [40]. This current paper is a continuation of this research project where data from Group 1 (control) were added for comparison with the GSR-BF rehabilitation group to demonstrate the effectiveness of the alternative treatment method.

BF training sessions were held twice a week, and standard rehabilitation sessions were held as specified in the ward's schedule. The schedule for the standard rehabilitation program contained rehabilitation exercises for every day of the week. An example of a day's schedule is as follows: Monday: 8.00–8.30 gymnastics, 9.00–10.00 breakfast, 10.30–11.00 community meeting, 11.30–12.30 classes in the art workshop, 13.00–14.00 lunch, 14.30–15.30 free time, 16.00–17.00 sport activities/walk, and 17.30–18.30 dinner.

Prior to therapy, the level of cognitive deficits (thinking, memory, concentration) was assessed using the CTT and d2 tests.

### 2.2. Statistical Analyses

The results of the measurements were analysed statistically. The Student's *t*-test for dependent samples, nonparametric Mann–Whitney *U*-test, and Spearman's rank correlation coefficient were used to compare results obtained before and after therapy. Differences were considered to be statistically significant at *p* < 0.05. The database was developed, and the statistical tests were performed using the Statistica 9.1 (StatSoft, Krakow, Poland) software.

### 2.3. Ethical Issues

The study protocol was approved by the local Bioethics Committee—approval no. KE-0254/35/2019. All the patients invited to take part in the study gave their written informed consent.

### 2.4. Patients Characteristics

Comparisons between the two groups showed that they did not differ statistically significantly in demographic and clinical characteristics such as age, education, place of residence, outpatient treatment, medication regimens, and suicide attempts. The mean age of Group 1 and Group 2 subjects was 36 years (*M* = 36.38SD = 8.87) and 37 years (*M* = 37.22SD = 6.38), respectively. In Group 1, one patient had primary education, six had vocational education, 13 had secondary education, and five had tertiary education. In Group 2, four patients had primary education, five had vocational education, and nine had secondary education. In Group 1, four patients were inhabitants of large cities, 10 lived in smaller towns, and 11 lived in the countryside. Most of the patients (14) in Group 2 lived in large cities of over 100,000 inhabitants, two lived in smaller towns (below 100,000 inhabitants), and two were country-dwellers. All subjects received atypical neuroleptics; in three patients from Group 1, they were administered via the IM route. Patients in both groups reported receiving irregular outpatient treatment (Group 1–6 people vs. Group 2–16 people) and no suicide attempts (Group 1–17 people vs. Group 2–11 people).

Small differences between the groups were found with regard to marital status, number of children, number of hospital admissions, employment, household composition, and family history of mental illness. There were 23 single men in Group 1 and 15 in Group 2. Similar numbers of patients in both groups reported having no children (Group 1–23 persons vs. Group 2–16 persons). The mean number of hospital admissions was also similar for the two groups (Group 1–8 vs. Group 2–6.8). The main source of income for patients in both groups was a disability pension (Group 1–16 persons vs. Group 2–12 persons), followed by odd jobs (Group 1–5 persons vs. Group 2–1 person) and social assistance benefits (Group 1–2 persons vs. Group 2–4 persons). Comparable numbers of respondents reported living with their parents (Group 1–21 persons vs. Group 2–13 persons). Also, similar numbers of patients had no family history of schizophrenia on the mother's side (Group 1–24 persons vs. Group 2–17 persons) or on the father's side of the family (Group 1–18 persons vs. Group 2–16 persons).

## 3. Results

To verify the assumptions made and evaluate the efficacy of GSR-BF therapy and standard rehabilitation in patients diagnosed with schizophrenia, the measurements were subjected to comparative analysis.  Table 1 presents only those results which showed statistically significant differences between measurements in both groups. The remaining differences were insignificant.

The analyses indicate that there were statistically significant differences between pretherapy and posttherapy measurements in both groups studied. In Group 1, statistically significant differences were found for the d2 test which showed a reduction in the number of errors the subjects made during the test (*M* = 9.0; SD = 10.9 vs. *M* = 6.3; SD = 7.0) and an improvement in their ability to concentrate (*M* = 107.4; SD = 46.7 vs. *M* = 117.9; SD = 35.7). In Group 2, statistically significant differences reflected an increase in the neurotrophic factor (*M* = 44.8; SD = 10.7 vs. *M* = 55.5; *SD* = 10.7) and improvements in reflectiveness on the BCISS scale (*M* = 22.7; SD = 4.8 vs. *M* = 25.7; SD = 3.1), illness acceptance on the AIS scale (*M* = 22.7; SD = 8.6 vs. *M* = 26.4; SD = 6.5), self-efficacy on the GSES scale (*M* = 23.8; SD = 5.4 vs. *M* = 27.6; SD = 5.1), and concentration, as demonstrated by the theta/beta (*M* = 2.1; SD = 0.6 vs. *M* = 2.3; SD = 0.9) and theta/SMR (*M* = 2.1; SD = 0.6 vs. *M* = 2.4; SD = 0.8) ratios and by evoked potentials, mainly the amplitude of the N100 wave (*M* = −3.6; SD = 2.5 vs. *M* = −5.4; SD = 1.9) and the latency of the P200 wave (*M* = 208.8; SD = 14.8 vs. *M* = 196.1; SD = 18.3). In both groups, statistically significant differences were noted for measurements on all PANSS subscales, which indicates that these two forms of rehabilitation had a similar therapeutic effect on the reduction of disease-related positive and negative symptoms.

As both GSR-BF and standard therapy led to statistically significant changes, an attempt was made in the further part of the study to determine which form of therapy was more effective. For this purpose, analyses were performed to show differences between the groups in the magnitude of change in the results obtained before and after rehabilitation. The analyses showed that the differences in the magnitude of change were statistically significant for only two variables. The data are presented in Table 2. Only significant differences are shown; other differences were not significant and therefore are not included.

*M*: mean; SD: standard deviation; A: Student's *t*-test; B: Mann–Whitney *U*-test; *p*: statistical significance.

For BDNF, a larger statistically significant difference was noted between measurements in Group 2 (*M* = 10.72; SD = 7.35) than in Group 1 (*M* = 2.80; SD = 8.9). Similarly, for GSES, the statistically significant difference between measurements was larger in Group 2 (*M* = 3.83; SD = 5.0) than in Group 1 (*M* = −1.46; SD = 7.5). For the remaining variables, no statistically significant differences were found in the magnitude of change in measurements; the magnitude of change in measurements in Group 1 was similar to the magnitude of change in Group 2. These analyses indicate that the individual parameters underwent similar changes, and the magnitude of changes achieved in the patients subjected to GSR-BF was similar to the magnitude of changes achieved in patients receiving standard rehabilitation.

Correlation analysis showed that in Group 1, standard rehabilitation exercises reduced the severity of positive and negative symptoms measured on the PANSS and improved the patients' attention and concentration (QEEG), as confirmed by the shortened P2 latency (Table 3).

Correlation analysis conducted in Group 2 showed that BF training reduced the severity of positive and negative symptoms measured on the PANSS, increased BDNF levels, improved attention and concentration (QEEG), and shortened P2 latency (Table 4).

## 4. Discussion

Technological progress and scientific research in various areas of medicine and engineering bring new solutions in the rehabilitation of mentally-ill patients. Currently, the focus is on neuronal mechanisms which, similarly to physiological markers, enable the correction of existing deficits. BF is a noninvasive method based on the feedback between the patient's mental condition and neurophysiological function which allows them to volitionally control their mental and physiological functions.

The study was aimed to compare two groups of male patients with a clinical diagnosis of schizophrenia, in the remission phase, who received two types of rehabilitation: standard rehabilitation (Group 1) vs. GSR-BF training (Group 2). The analyses indicate that in both Group 1 and Group 2 there were statistically significant differences between pretherapy and posttherapy measurements on the PANSS scale, which reflected a reduction in disease-related positive and negative symptoms. The results show that rehabilitation had a positive effect in both groups of patients, regardless of the method of rehabilitation used.

In Group 1, statistically significant differences were found for the d2 test, which indicated a reduction in the number of mistakes the subjects made during the test and an improvement in their ability to concentrate. Also in Group 2, there was a statistically significant improvement in concentration, as confirmed by the theta/beta and theta/SMR ratios, and an improvement in the initial perceptual analysis, as disclosed by the N1 wave amplitude and the P2 wave latency [41]. Additionally, in Group 2, there was a statistically significant increase in BDNF, and an increase in reflectiveness, illness acceptance, and self-efficacy.

Further analyses of statistically significant differences between the groups in the magnitude of change in the results obtained before and after rehabilitation also showed that the two forms of therapy had a similar effect. Comparable effects were observed for nearly all dependent variables, except for BDNF and self-efficacy, which improved noticeably more in patients undergoing GSR-BF therapy compared to the patients in the standard rehabilitation program. Comparative analyses demonstrated that both forms of rehabilitation are effective and can be applied alternately.

The effect of GSR-BF therapy seems to be especially interesting, as training led to improvement in both the subjects' cognitive and social functioning. This outcome was probably related to the modulation of brain activity. People subjected to BF training learn how to modulate the bioelectrical activity of their brain in accordance with their own expectations. The important point is that no complicated equipment is required, and the method is practical and simple to apply, when compared to other neuromodulation techniques. Some studies confirm that the effect of BF therapy can be maintained for prolonged periods of time [42, 43].

Numerous reports indicate that cognitive training through a brain–computer interface enables modification of the bioelectrical activity of the brain in patients with various mental disorders, including those diagnosed with schizophrenia, and repeated stimulation has a positive effect not only on stimulus–response components but also on the change in the intensity of interneuronal connections and an increase in the number of synaptic connections [42, 44, 45]. This was proven in an experiment in which individual components of evoked potentials showed specific changes in the ERP recording through positive and negative polarisation. The shape of that recording was associated with the influence of the stimulus presented to the subjects on their behavioural response [46]. It can be assumed that the component was an indicator of cognitive processes and reflected brain activity [47]. In this study, this was also confirmed by the stimulus compatibility effect and the increase in BDNF. The elevated levels of this neurotrophic factor were possibly caused by the increase in the interplanar transfer of information [48].

Similar results were obtained by Iwata et al. [49], who compared the effects of standard rehabilitation and training using a computer application (Cog Pack). Although both types of intervention improved the patients' cognitive function, the group training with the computer application achieved a significantly greater improvement in the speed of information processing and performance functions, as confirmed by the Brief Assessment of Cognition in Schizophrenia (BACS) and the Life Assessment Scale for the Mentally Ill (LISMI).

It is worth emphasising that cognitive functions, such as perception, attention, and memory, are correlated with synchronous oscillations, which generate the theta rhythm in the neuronal networks of the hippocampus through the cooperation of two neurotransmission systems: cholinergic and GABA-ergic, thus inducing neuroplastic changes at the synaptic level, so-called long-term synaptic strengthening and memory trances [45, 50].

For such process to be induced, QEEG ranges must undergo a detailed analysis, and the sequences of all brain regions must be taken into account versus relevant standards. QEEG analysis allows to develop training protocols (mainly in EEG BF therapy) and a variety of exercises to enable a reduction in hypercoherence which indicates that the brain function is not differentiated, and its functional “flexibility” is limited. An example here can be a study of 51 pharmacotherapy naive people diagnosed with schizophrenia who underwent QEEG evaluation. The analysis showed that in all study participants, the bioelectrical function of the brain was similar to the brain function in people with chronic schizophrenia. By establishing appropriate protocols and planning EEG-BF training, the researchers achieved a statistically significant reduction in positive and negative symptoms of the disease on the PANSS (20% improvement). After a series of training sessions, the brain bioelectrical function of 19 patients differed significantly from the function in patients diagnosed with chronic schizophrenia [51].

Real-time functional magnetic resonance imaging (rt-fMRI) was used for the first time in 1995, and evidence for the usefulness of this method in neurorehabilitation was provided in 2005 [52]. rt-fMRI scans confirmed changes in targeted neuronal networks already after a single 30-minute EEG-BF session [53], and after numerous sessions, the scans revealed changes in specific regions related to symptoms [54]. This evaluation was possible owing to simultaneous verification by rt-fMRI and EEG-BF, in the recording of which the spatial resolution of fMRI and the time resolution of EEG were used [55].

In 2013, rt-fMRI was used in a study of schizophrenia patients who were trained to regulate the response of the frontal insular cortex using EEG BF. The goal of the experiment was to demonstrate a relationship between EEG-BF training, recognising facial emotions, and insular activation. The subjects showed a significant improvement in the recognition of disgust, which was associated with the activation of the frontal insula, and an increased number of incoming and outgoing connections. That study was the first to demonstrate that rt-fMRI EEG-BF could be used to teach schizophrenia patients to volitionally regulate their brain activity [56]. In another study, an attempt was made to improve cognitive functions in schizophrenia patients by rt-fMRI EEG-BF training of the frontal cingulate gyrus as a structure significantly involved in cognitive processes. In this experiment, EEG-BF training resulted in the activation of the dorsal part of the frontal cingulate gyrus in the schizophrenia subjects and the activation of its ventral part in control subjects. Functionally, the dorsal part of the frontal cingulate gyrus is activated in cognitive tasks, while the ventral part is activated in emotional processes. Those authors concluded that rt-fMRI BF offered an opportunity to directly influence the neural network, with simultaneous monitoring of the effects of that influence [57, 58].

Although the test results reported in this present study concern GSR-BF training (without protocols applied), the demonstrated therapeutic effect and QEEG data (pre- and posttherapy) confirm the results obtained by other authors. The ability to transform behavioural states into underlying brain dynamics is very useful [43, 59], and the rehabilitation interventions based on this mechanism play a great role in the improvement of those states [57, 60, 61].

There are some limitations of this study which should be taken into account considering its results. EEG was performed in every patient qualified in accordance with the criteria for research in order to exclude neurological diseases. QEEG was performed twice, at the beginning of the experiment and after three months (after both types of rehabilitation). The limitation of the study may be the lack of the first QEEG screening test. The authors decided that the first examination would be the general starting parameter for the study. Additional limitation is a sample size; further study is recommended on a bigger study sample.

## 5. Conclusions

1. The scale of changes achieved in the group of patients subjected to GSR-BF therapy was similar to the scale of changes achieved in patients subjected to standard rehabilitation. However, experimental rehabilitation based on neurophysiological GSR-Biofeedback training confirms the improvement of cognitive and social functioning of the subjects. In the cognitive area, it is proved by a decrease in the intensity of psychopathological symptoms (positive and negative) and an improvement in attention, concentration, and initial stimulus analysis. In the social area, it is confirmed by reduction of internal tension and increase of self-efficacy of the respondents. Additionally, an increase in the neurotrophic factor BDNF, which as an indicator of neuromodulation justifies the occurring neurophysiological changes
2. GSR-BF can be used as a new form of therapeutic intervention in patients diagnosed with schizophrenia and represents an alternate approach to standard rehabilitation

## Figures and Tables

**Table 1:** Variables which showed statistically significant differences between pretherapy and posttherapy measurements in both study groups.

Variable	Group	Examination I (before)		Examination II (after)		Difference	Difference significance		Confidence level	
		*M*	SD	*M*	SD		*T*	*p*	−95%	+95%
d2.%B (errors)	2	10.70	11.09	8.71	10.33	−1.99	0.741	0.471	−7.74	3.77
	1	9.01	10.89	6.25	7.01	2.76	2.107	0.046	0.05	5.47
d2. ZK (ability to concentrate)	2	99.06	44.59	105.94	47.66	6.88	−0.985	0.340	−8.00	21.75
	1	107.42	46.69	117.88	35.71	−10.46	−2.078	0.049	−20.87	−0.05
PANSS-POSITIVE	2	9.06	2.04	7.50	2.23	−1.56	10.719	<0.001	−1.86	−1.25
	1	9.28	2.01	8.24	2.01	1.04	6.186	<0.001	0.69	1.39
PANSS-NEGATIVE	2	13.94	3.92	11.83	4.48	−2.11	8.304	<0.001	−2.65	−1.57
	1	15.16	3.51	14.08	4.47	1.08	2.596	0.016	0.22	1.94
PANSS-GENERAL	2	24.83	3.35	22.61	3.71	−2.22	10.736	<0.001	−2.66	−1.79
	1	27.44	3.31	25.88	4.20	1.56	2.742	0.011	0.39	2.73
PANSS-TOTAL	2	47.83	8.49	41.94	9.64	−5.89	11.834	<0.001	−6.94	−4.84
	1	51.92	7.22	48.20	9.36	3.72	3.375	0.003	1.45	6.00
BDNF	2	44.78	10.69	55.50	10.76	10.72	−6.185	<0.001	7.06	14.38
	1	50.16	11.38	52.96	10.70	−2.80	−1.575	0.128	−6.47	0.87
BCIS A (self-reflectiveness)	2	22.72	4.80	25.72	3.14	3.00	−3.170	0.006	−5.00	−1.00
	1	21.15	4.47	22.12	4.96	−0.96	−0.911	0.371	−3.14	1.21
BCISS A-B (composite index)	2	8.78	5.35	12.22	3.17	3.44	−2.946	0.009	−5.91	−0.98
	1	6.38	4.83	7.35	5.12	−0.96	−1.000	0.327	−2.94	1.02
AIS (illness acceptance)	2	22.67	8.95	26.44	6.46	3.78	−2.547	0.021	0.65	6.91
	1	25.96	8.77	25.00	7.83	0.96	0.557	0.583	−2.60	4.52
GSES (self-efficacy)	2	23.78	5.43	27.61	5.09	3.83	−3.239	0.005	1.34	6.33
	1	30.15	5.76	28.69	6.16	1.46	1.000	0.327	−1.55	4.47
QEEG C-z theta/beta (attention factor of the central area)	2	1.92	0.57	2.29	0.88	0.37	−2.632	0.018	0.07	0.67
	1	2.35	0.94	2.49	0.82	−0.14	−1.453	0.159	−0.34	0.06
QEEG F-z theta/SMR (concentration factor of the central area)	2	2.07	0.64	2.37	0.80	0.30	−2.358	0.031	0.03	0.57
	1	2.49	1.00	2.60	0.83	−0.10	−1.013	0.321	−0.31	0.10
F-z N1 (amplitude of the first negative component of the central area)	2	−3.95	2.53	−5.36	1.93	−1.41	2.588	0.020	−2.57	−0.26
	1	−5.29	3.93	−6.58	3.44	1.30	1.263	0.219	−0.83	3.42
C-z P2 (latency—delay of the second positive component of the central area)	2	208.82	14.81	196.06	18.27	−12.77	2.643	0.018	−23.01	−2.52
	1	203.92	23.94	205.04	21.70	−1.13	−0.185	0.855	−13.68	11.43

M: mean value; SD: standard deviation; T: Student's *t*-test; *p*: level of significance.

**Table 2:** Statistically significant differences between groups in the magnitude of change from pretherapy to posttherapy measurements.

Variable (change between measurements for the variable)	Group 1		Group 2		Comparison between groups	
	*M*	SD	*M*	SD	t^A^/U^B^	*p*
BDNF (neurotrophic factor)	2.80	8.89	10.72	7.35	−3.093^A^	0.004
GSES (self-efficacy)	−1.46	7.45	3.83	5.02	119.5^B^	0.005

**Table 3:** Correlations between the magnitude of changes from pretherapy to posttherapy measurements in the group of patients following a standard rehabilitation program (Group 1).

Variable	Group 1 (standard rehabilitation program)								
	PANSS POS	PANSS NEG	PANSS GEN	PANSS TOT	BDNF (ng/m)	QEEG theta/beta	QEEG theta/SMR	N1 amplitude	P2 latency
PANSS-POSITIVE	—	0.315	0.588∗	0.712∗	−0.211	0.034	0.078	0.193	−0.405
PANSS-NEGATIVE	0.315	—	0.568∗	0.799∗	−0.343	0.388	0.399	−0.028	−0.100
PANSS-GENERAL	0.588^∗^	0.568^∗^	—	0.880^∗^	−0.085	0.038	0.042	0.272	−0.030
PANSS-TOTAL	0.712^∗^	0.799^∗^	0.880^∗^	—	−0.221	0.147	0.168	0.192	−0.174
BDNF(ng/ml)	−0.211	−0.343	−0.085	−0.221	—	0.101	0.140	0.433	−0.117
QEEG theta/beta	0.034	0.388	0.038	0.147	0.101	—	0.904^∗^	0.007	−0.498^∗^
QEEG theta/SMR	0.078	0.399	0.042	0.168	0.14	0.904^∗^	—	0.181	−0.488^∗^
N1 (amplitude)	0.193	−0.028	0.272	0.192	0.433	0.007	0.181	—	−0.555^∗^
P2 (latency)	−0.405	−0.100	−0.030	−0.174	−0.117	−0.498^∗^	−0.488^∗^	−0.555^∗^	—

Legend: correlations were assessed using Spearman's rank correlation coefficients (italics) and Pearson's *r*; statistically significant correlations (*p* < 0.050) are marked with an asterisk (^∗^).

**Table 4:** Correlations between the magnitude of changes from pretherapy to posttherapy measurements in the group of patients participating in GSR-BF training sessions (Group 2).

Variable	Group 2 (BF training program)								
	PANSS POS	PANSS NEG	PANSS GEN	PANSS TOT	BDNF (ng/ml)	QEEG theta/beta	QEEG theta/SMR	N1 ampl.	P2 latency
PANSS-POSITIVE	—	0.737^∗^	0.851^∗^	0.877^∗^	−0.770^∗^	0.171	0.274	−0.106	0.074
PANSS-NEGATIVE	0.737^∗^	—	0.846^∗^	0.920^∗^	−0.857^∗^	0.004	0.018	−0.228	−0.061
PANSS-GENERAL	0.851^∗^	0.846^∗^	—	0.956^∗^	−0.804^∗^	0.112	0.169	−0.103	0.172
PANSS-TOTAL	0.877^∗^	0.920^∗^	0.956^∗^	—	−0.832^∗^	0.149	0.209	−0.166	0.061
BDNF (ng/ml)	−0.770^∗^	−0.857^∗^	−0.804^∗^	−0.832^∗^	—	0.123	0.057	0.153	0.296
QEEG theta/beta	0.171	0.004	0.112	0.149	0.123	—	0.875^∗^	−0.161	−0.127
QEEG theta/SMR	0.274	0.018	0.169	0.209	0.057	0.875^∗^	—	−0.298	−0.297
N1 (amplitude)	−0.106	−0.228	−0.103	−0.166	0.153	−0.161	−0.298	—	0.035
P2 (latency)	0.074	−0.061	0.172	0.061	0.296	−0.127	−0.297	0.035	—

Legend: correlations were assessed using Spearman's rank correlation coefficients (italics) and Pearson's *r*; statistically significant correlations (*p* < 0.050) are marked with an asterisk (^∗^).

## Data Availability

Available at authors on request.
